# An Advance Computing Numerical Heuristic of Nonlinear SIR Dengue Fever System Using the Morlet Wavelet Kernel

**DOI:** 10.1155/2022/9981355

**Published:** 2022-01-31

**Authors:** Muhammad Umar, Zulqurnain Sabir, Muhammad Asif Zahoor Raja, K. S. Al-Basyouni, S. R. Mahmoud, Yolanda Guerrero Sánchez

**Affiliations:** ^1^Department of Mathematics and Statistics, Hazara University, Mansehra, Pakistan; ^2^Future Technology Research Center, National Yunlin University of Science and Technology, 123 University Road, Section 3, Douliou, Yunlin 64002, Taiwan; ^3^Mathematics Department, Faculty of Science, King Abdulaziz University, Jeddah, Saudi Arabia; ^4^GRC Department, Faculty of Applied Studies, King Abdulaziz University, Jeddah, Saudi Arabia; ^5^Department of Dermatology, Stomatology, Radiology and Physical Medicine, University of Murcia, Murcia, Spain

## Abstract

This study is associated to solve the nonlinear SIR dengue fever system using a computational methodology by operating the neural networks based on the designed Morlet wavelet (MWNNs), global scheme as genetic algorithm (GA), and rapid local search scheme as interior-point algorithm (IPA), i.e., GA-IPA. The optimization of fitness function based on MWNNs is performed for solving the nonlinear SIR dengue fever system. This MWNNs-based fitness function is accessible using the differential system and initial conditions of the nonlinear SIR dengue fever system. The designed procedures based on the MWNN-GA-IPA are applied to solve the nonlinear SIR dengue fever system to check the exactness, precision, constancy, and efficiency. The achieved numerical form of the nonlinear SIR dengue fever system via MWNN-GA-IPA was compared with the Runge–Kutta numerical results that verify the significance of MWNN-GA-IPA. Moreover, statistical reflections through different measures for the nonlinear SIR dengue fever system endorse the precision and convergence of the computational MWNN-GA-IPA.

## 1. Introduction

Dengue fever disease (DFD) is one of the epidemics, infectious, and serious diseases that disturbed about 2.5 billion individuals all over the world. DFD occurred in some main countries of Southeast Asia due to the hot seasons. The infectious DFD grows fast, when the environment alters and becomes dangerous because of the shortage of information amongst the individuals [1]. DFD is an epidemiologic transmittable fever formed by dengue infection (DI) that is conveyed through mosquitoes to humans and apes [2]. Some symptoms scientifically produced by DFD are headache, joint pain, skin rash, and DI. The global World Health Organization (WHO) classified DI into a hemorrhagic dengue fever before one decade [3]. DI is categorized into three organizational proteins, membrane protein (M), envelope protein (E), and capsid protein (C), while it has seven proteins that are nonstructural and their names are NS-I, NS-IIA, NS-III, NS-IIB, NS-IVA, NS-IVB, and NS-V [4]. According to envelope protein antigenicity, DI is ordered into four classes of microorganisms, which are infected as well as pathogenic [5].

DI has been reported in several zones of China and still any scientific report cannot prove it a confined endemic [6], whereas all other subgroups of DI have been imported; DI-I and DI-II are considered in China one of the main stereotypes endemic. In the Chinese province Guangdong, DV-I reported around 70% in 2014 and 80% in 2015. Presently, an amino-based acid localizes transformation in NS-I of the Asian “Zika” inheritance, which has been described to grow the production of NS-I in the diseased host to make the virus convenient to Aedes type of mosquitoes, which is the focal wide spreading cause of virus “Zika” since 2015 [7].

Some epidemic infections such as COVID-19 are the existing transferred diseases, which have covered the whole world and the infection rate along with the number of deaths from COVID-19 increased steadily [8]. Another common disease is malaria, which is not directly transmitted from host to host. Protozoa is one of the transferred diseases, which spreads due to the anopheles of the female mosquito. According to the WHO report, almost 1/3 million individuals per year die from malaria. It distresses the children and pregnant women, mostly in the South African and American countries. Many chemical sprays have been widely implemented to control the mosquito population. Similarly, nonpolluting types of biological arrangements normally accomplished to emphasis the ecosystem of complicated kinds. The sterile insect apparatus (SIA) is a proficient nonpolluting scheme of insect control, which depends on the sterile male's release. Consequently, adequately sterile males discharging causes the elimination of the wild's population. Over a half century ago, SIA has been recognized in the Curacao Island to adjust the screwworm hover [9, 10].

The aim of this study is to solve the nonlinear SIR dengue fever system using a computational methodology by operating the MWNNs, global search GA, and rapid local search IPA, i.e., MWNN-GA-IPA. The stochastic approaches have been investigated normally to solve a number of applications directed to the differential linear/nonlinear systems [11, 12]. However, no one has applied the MWNNs to solve the nonlinear SIR dengue fever system. Few recent reported submissions of stochastic solvers are eye surgery model, functional singular system, Thomas–Fermi singular equation, HIV-based infection system, biological form of the prey-predator system, periodic singular problems, singular three-point differential model, COVID-19 SITR system, multifractional singular models, system of heat transmission in human head, and mosquito spreading in heterogeneous conditions [13–15]. The intention of this study is to solve the nonlinear SIR dengue fever system using the MWNN-GA-IPA. The literature form of nonlinear SIR dengue fever system is written as [16]

(1) $$\begin{array}{c} \left\{\begin{array}{cc} \frac{\text{d}X\left(\tau \right)}{\text{d}\tau }=\mu_{h}-\mu_{h}X\left(\tau \right)-\alpha X\left(\tau \right)Z\left(\tau \right), & X\left(0\right)=I_{1},\\ \frac{\text{d}Y\left(t\right)}{\text{d}\tau }=\alpha X\left(\tau \right)Z\left(\tau \right)-\beta Y\left(\tau \right), & Y\left(0\right)=I_{2},\\ \frac{\text{d}Z\left(t\right)}{\text{d}\tau }=\gamma Y\left(\tau \right)-\gamma Y\left(\tau \right)Z\left(\tau \right)-\delta_{1}Z\left(\tau \right), & Z\left(0\right)=I_{3}, \end{array}\right. \end{array}$$

where the susceptible class, infected class, and recovered class are *X*(*τ*), *Y*(*τ*), and *Z*(*τ*), respectively. The terms *γ*, *μ*_*h*_, *δ*_1_, *α*, and *β* used in system (1) are constant, whereas the initial conditions are *I*_1_, *I*_2_, and *I*_3_, respectively. Few major geographies of the MWNN-GA-IPA are concisely given as follows:

- Design of Morlet wavelet is presented successfully as an activation function to solve the nonlinear SIR dengue fever system
- The reliable, consistent, and stable overlapped results obtained by the MWNN-GA-IPA and the true solutions validate the exactness of the proposed approach
- The authentication of the presentation is trained via different statistical valuations to get the solutions of the nonlinear SIR dengue fever system on multiple executions of the MWNN-GA-IPA

The rest of this paper is reported as follows: Section 2 indicates the proposed MWNN-GA-IPA along with the statistical measures.  Section 3 shows the results simulations.  Section 4 describes the final remarks and future research reports.

## 2. Designed Procedure

The proposed structure of the MW-GA-IPA is used to solve the nonlinear SIR dengue fever system described in two phases as follows:

- An objective function using the MW is considered to activate the neural networks
- Necessary clarifications are provided to enhance the merit function by applying the hybrid of GA-IPA

### 2.1. Designed Procedure Using MW Function

The mathematical design of the nonlinear SIR dengue fever system is described by using the achieved results of susceptible $\hat{X}\left(\tau \right)$, infected $\hat{Y}\left(\tau \right)$, and recovered $\hat{Z}\left(\tau \right)$ with the derivatives of these classes, written as [17]

(2) $$\begin{array}{c} \left[\hat{X}\left(\tau \right),\hat{Y}\left(\tau \right),\hat{Z}\left(\tau \right)\right]=\left[\begin{array}{c} \sum_{i=1}^{m}v_{X,i}H\left(w_{X,i}\tau +u_{X,i}\right),\sum_{i=1}^{m}v_{Y,i}H\left(w_{Y,i}\tau +u_{Y,i}\right),\\ \sum_{i=\;1}^{m}v_{Z,i}H\left(w_{Z,i}\tau +u_{Z,i}\right) \end{array}\right],\\ \left[{\hat{X}}^{\left(n\right)}\left(\tau \right),{\hat{Y}}^{\left(n\right)}\left(\tau \right),{\hat{Z}}^{\left(n\right)}\left(\tau \right)\right]=\left[\begin{array}{c} \sum_{i=1}^{m}v_{X,i}H^{\left(n\right)}\left(w_{X,i}\tau +u_{X,i}\right),\sum_{i=1}^{m}v_{Y,i}H^{\left(n\right)}\left(w_{Y,i}\tau +u_{Y,i}\right),\\ \sum_{i=1}^{m}v_{Z,i}H^{\left(n\right)}\left(w_{Z,i}\tau +u_{Z,i}\right) \end{array}\right], \end{array}$$

***W*** is the unknown weight vector given as **W**=[**W**_*X*_; **W**_*Y*_; **W**_*Z*_], for **W**_*X*_=[**v**_*X*_,*ω*_*X*_, **u**_*X*_], **W**_*Y*_=[**v**_*Y*_,*ω*_*Y*_, **u**_*Y*_], and **W**_*Z*_=[**v**_*Z*_,*ω*_*Z*_, **u**_*Z*_], where

(3) $$\begin{array}{c} v_{X}=\left[v_{X,1};\;v_{X,2};\;\ldots ;\;v_{X,m}\right],\;v_{Y}=\left[v_{Y,1};\;v_{Y,2};\;\ldots ;v_{Y,m}\right],\;v_{Z}=\left[v_{Z,1};\;v_{Z,2};\;\ldots ;\;v_{Z,m}\right],\\ w_{X}=\left[w_{X,1};\;w_{X,2};\;\ldots ;\;w_{X,m}\right],\;w_{Y}=\left[w_{Y,1};\;w_{Y,2};\;\ldots ;\;w_{Y,m}\right],\;w_{Z}=\left[w_{Z,1};\;w_{Z,2};\;\ldots ;\;w_{Z,m}\right],\\ u_{X}=\left[u_{X,1};\;u_{X,2};\;\ldots ;u_{X,m}\right],\;u_{Y}=\left[u_{Y,1};\;u_{Y,2};\;\ldots ;\;u_{Y,m}\right],\;u_{Z}=\left[u_{Z,1};\;u_{Z,2};\;\ldots ;\;u_{Z,m}\right]. \end{array}$$

The MWNN has not been implemented before to solve the nonlinear SIR dengue fever system. The mathematical form of MW function is written as [18]

(4) $$\begin{array}{c} H\left(\tau \right)=\cos\left(1.75\right)e^{-0.5\tau^{2}}. \end{array}$$

The simplified form of system (2) using the above MW function is given as

(5) $$\begin{array}{c} \left[\hat{X}\left(\tau \right),\hat{Y}\left(\tau \right),\hat{Z}\left(\tau \right)\right]=\left[\begin{array}{c} \sum_{i=1}^{m}v_{X,i}\cos\left(1.75\left(w_{X,i}\tau +u_{X,i}\right)\right)e^{-0.5{\left(w_{X,i}\tau +u_{X,i}\right)}^{2}},\\ \sum_{i=1}^{m}v_{Y,i}\cos\left(1.75\left(w_{Y,i}\tau +u_{Y,i}\right)\right)e^{-0.5{\left(w_{Y,i}\tau +u_{Y,i}\right)}^{2}},\\ \sum_{i=1}^{m}v_{Z,i}\cos\left(1.75\left(w_{Z,i}\tau +u_{Z,i}\right)\right)e^{-0.5{\left(w_{Z,i}\tau +u_{Z,i}\right)}^{2}}, \end{array}\right],\\ \left[{\hat{X}}^{\left(n\right)}\left(\tau \right),{\hat{Y}}^{\left(n\right)}\left(\tau \right),{\hat{Z}}^{\left(n\right)}\left(\tau \right)\right]=\frac{d}{\text{d}\tau }\left[\begin{array}{c} \sum_{i=1}^{m}v_{X,i}\cos\left(1.75\left(w_{X,i}\tau +u_{X,i}\right)\right)e^{-0.5{\left(w_{X,i}\tau +u_{X,i}\right)}^{2}},\\ \sum_{i=1}^{m}v_{Y,i}\cos\left(1.75\left(w_{Y,i}\tau +u_{Y,i}\right)\right)e^{-0.5{\left(w_{Y,i}\tau +u_{Y,i}\right)}^{2}},\\ \sum_{i=1}^{m}v_{Z,i}\cos\left(1.75\left(w_{Z,i}\tau +u_{Z,i}\right)\right)e^{-0.5{\left(w_{Z,i}\tau +u_{Z,i}\right)}^{2}}. \end{array}\right]. \end{array}$$

An error function based on the merit function is given as

(6) $$\begin{array}{c} e=\sum_{j=i}^{4}e_{j}, \end{array}$$

(7) $$\begin{array}{c} e_{1}=\frac{1}{N}\sum_{i=1}^{N}{\left[{\hat{X^{\prime }}}_{i}-\mu_{h}+\mu_{h}{\hat{X}}_{i}+\alpha {\hat{X}}_{i}{\hat{Z}}_{i}\right]}^{2}, \end{array}$$

(8) $$\begin{array}{c} e_{2}=\frac{1}{N}\sum_{i=1}^{N}{\left[{{\hat{Y}}^{\prime }}_{i}-\alpha {\hat{X}}_{i}{\hat{Z}}_{i}+\beta {\hat{Y}}_{i}\right]}^{2}, \end{array}$$

(9) $$\begin{array}{c} e_{3}=\frac{1}{N}\sum_{i=1}^{N}{\left[{{\hat{Z}}^{\prime }}_{i}-\gamma {\hat{Y}}_{i}+\gamma {\hat{Z}}_{i}{\hat{Y}}_{i}+\delta_{1}{\hat{Z}}_{i}\right]}^{2}, \end{array}$$

(10) $$\begin{array}{c} e_{4}=\frac{1}{3}\left[{\left({\hat{X}}_{0}-I_{1}\right)}^{2}+{\left({\hat{Y}}_{0}-I_{2}\right)}^{2}+{\left({\hat{Z}}_{0}-I_{3}\right)}^{2}\right], \end{array}$$

where ${\hat{X}}_{i}=X\left(\tau_{i}\right),\;{\hat{Y}}_{i}=\hat{Y}\left(\tau_{i}\right),\;{\hat{Z}}_{i}=Z\left(\tau_{i}\right),\;Nh=1,$ and *τ*_*i*_=*ih*. ${\hat{X}}_{i}$, ${\hat{Y}}_{i}$ and ${\hat{Z}}_{i}$ show the proposed results of the susceptible class, infected class, and recovered class. Likewise, *e*_1_, *e*_2_, and *e*_3_ denote the error function related to system (1), whereas *e*_4_ denotes the error function on the basis of initial conditions.

### 2.2. Optimization: MWNN-GA-IPA

The optimization performance is presented for solving the nonlinear SIR dengue fever system using the MWNN-GA-IPA. The structure of the present approach to solve the nonlinear SIR dengue fever system is provided in Figure 1.

GA is a global optimization procedure, which is executed to solve the nonlinear SIR dengue fever system by implementing the usual selection procedures. GA is pragmatic frequently to regulate the accurate population to solve several complicated or stiff systems. To attain the best model outcomes, GAs operate through the operators based on selection, reproduction, crossover, and mutation. Few existing GA's applications are the hospitalization expenditure system [19], feature assortment in cancer microarray [20], organization of irregular magnetic character brain tumor imageries [21], vehicle routing system [22], prediction-based traffic flow system [23], radiation shielding optimizations in the bismuth-borate spectacles [24], prediction of air blast [25], composition optimization of cloud service [26], task arrangement models in phased range radar [27], arrangement system of microarray cancer [28], system dynamics of monorail vehicle [17], and prediction system of liver disease [29].

IPA is known as an optimized local search approach, which is performed broadly in both types of models (constrained/unconstrained). IPA is used in the optimization of various complicated and nonstiff natured systems. Recently, IPA is executed for image restoration [30], multistage nonlinear nonconvex models [31], viscoplastic fluid flows [32], nonsmooth contact dynamics [33], power systems [34], and dynamic flux balance analysis models [35]. The hybridization process of GA-IPA is applied to remove the laziness of GA, i.e., global approach. The pseudocode based on the designed approach MWNN-GA-IPA is provided in Table 1.

### 2.3. Performance Measures

The mathematical measures using the statistical operators for variance accounted for (VAF), semi-interquartile (S.I) range, Theil's inequality coefficient (T.I.C), and mean absolute deviation (M.A.D) along with the Global VAF (G-VAF), Global M.A.D (G-M.A.D), and Global T.I.C to solve the nonlinear SIR dengue fever system which is given as

(11) $$\begin{array}{c} \left\{\begin{array}{c} \left[\text{V.A}{\text{.F}}_{X},\text{ V.A}{\text{.F}}_{Y},\text{ V.A}{\text{.F}}_{Z}\right]=\left[\begin{array}{c} \left(1-\frac{\mathrm{var}\left(X_{r}-{\hat{X}}_{r}\right)}{\mathrm{var}\left(X_{r}\right)}\right)*100,\left(1-\frac{\mathrm{var}\left(Y_{r}-{\hat{Y}}_{r}\right)}{\mathrm{var}\left(Y_{r}\right)}\right)*100,\\ \left(1-\frac{\mathrm{var}\left(Z_{r}-{\hat{Z}}_{r}\right)}{\mathrm{var}\left(Z_{r}\right)}\right)*100, \end{array}\right]\\ \left[\text{E}-\text{V.A}{\text{.F}}_{X},\text{ E}-\text{V.A}{\text{.F}}_{Y},\text{ E}-\text{V.A}{\text{.F}}_{Z}\right]=\left[\left|100-\text{V.A}{\text{.F}}_{X},\;100-\text{V.A}{\text{.F}}_{Y},\;100-\text{V.A}{\text{.F}}_{Z}\right|\right]. \end{array}\right., \end{array}$$

(12) $$\begin{array}{c} \left\{\begin{array}{c} \text{S.I Range}=-0.5\times \left(Q_{1}-Q_{3}\right),\\ Q_{1}=\;1^{\text{st}}\text{ quartile \& }Q_{1}\;=3^{\text{rd}}\text{ quartile,} \end{array}\right., \end{array}$$

(13) $$\begin{array}{c} \left[\text{T.I}{\text{.C}}_{X},\text{T.I}{\text{.C}}_{Y},\text{T.I}{\text{.C}}_{Z}\right]=\left[\begin{array}{c} \frac{\sqrt{\left(1/n\right)\sum_{r=1}^{n}{\left(X_{r}-{\hat{X}}_{r}\right)}^{2}}}{\left(\sqrt{\left(1/n\right)\sum_{r=1}^{n}X_{r}^{2}}+\sqrt{\left(1/n\right)\sum_{r=1}^{n}{\hat{X}}_{r}^{2}}\right)},\frac{\sqrt{\left(1/n\right)\sum_{r=1}^{n}{\left(Y_{r}-{\hat{Y}}_{r}\right)}^{2}}}{\left(\sqrt{\left(1/n\right)\sum_{r=1}^{n}Y_{r}^{2}}+\sqrt{\left(1/n\right)\sum_{r=1}^{n}{\hat{Y}}_{r}^{2}}\right)},\\ \frac{\sqrt{\left(1/n\right)\sum_{r=1}^{n}{\left(Z_{k}-{\hat{Z}}_{k}\right)}^{2}}}{\left(\sqrt{\left(1/n\right)\sum_{r=1}^{n}{\hat{Z}}_{r}^{2}}+\sqrt{\left(1/n\right)\sum_{r=1}^{n}{\hat{Z}}_{r}^{2}}\right)}, \end{array}\right], \end{array}$$

where the approximate solutions are $\hat{X}$, $\hat{Y}$, and $\hat{Z}$, respectively.

## 3. Simulations of the Results

The current work is associated to solve the nonlinear SIR dengue fever system shown in system (1). The relative presentation of the obtained results using the Runge–Kutta solutions is tested to form the correctness of MWNN-GA-IPA. Additionally, statistical operators indicate the precision and accuracy of MWNN-GA-IPA. The simplified measures of the nonlinear SIR dengue fever system using the suitable values are given as

(14) $$\begin{array}{c} \left\{\begin{array}{cc} \hat{X^{\prime }}\left(\tau \right)=0.000046-\left(0.000046+0.375Z\left(\tau \right)\right)X\left(\tau \right), & X\left(0\right)=0.9999,\\ \hat{Y^{\prime }}\left(\tau \right)=0.375X\left(\tau \right)Z\left(\tau \right)-0.0323Y\left(\tau \right) & Y\left(0\right)=0.0006,\\ \hat{Z^{\prime }}\left(\tau \right)=0.328833-\left(0.328833Y\left(\tau \right)+0.0001\right)Z\left(\tau \right), & Z\left(0\right)=0.0560. \end{array}\right. \end{array}$$

The fitness function for system (14) is written as

(15) $$\begin{array}{c} e=\frac{1}{N}\sum_{i=1}^{N}\left(\begin{array}{c} {\left[{\hat{X^{\prime }}}_{r}-\left(0.000046+0.375{\hat{Z}}_{r}\right){\hat{X}}_{r}\right]}^{2}+{\left[{{\hat{Y}}^{\prime }}_{r}-0.375{\hat{X}}_{r}{\hat{Z}}_{r}+0.0323{\hat{Y}}_{r}\right]}^{2}\\ +{\left[{{\hat{Z}}^{\prime }}_{r}-\left(0.328833{\hat{Y}}_{r}+0.0001\right){\hat{Z}}_{r}\right]}^{2} \end{array}\right)\\ +\frac{1}{3}\left[{\left({\hat{X}}_{0}-\frac{9999}{10000}\right)}^{2}+{\left({\hat{Y}}_{0}-\frac{6}{10000}\right)}^{2}+{\left({\hat{Z}}_{0}-\frac{56}{1000}\right)}^{2}\right]. \end{array}$$

The nonlinear SIR dengue fever system given in system (1) is optimized using the MWNN-GA-IPA for 100 trials to attain ANN model parameters for 10 neurons. Figure 1 is drawn using the best outputs of the weight vector, i.e., ***W*** for the MWNN-GA-IPA. These best weights of the output are applied to solve the estimated outcomes of the nonlinear SIR dengue fever system. The mathematical illustrations of these estimated results from MWNN-GA-IPA are given as

(16) $$\begin{array}{c} \hat{X}\left(\tau \right)=0.067\;\cos\left(1.75\left(0.2561\tau -0.2972\right)\right)e^{-0.5{\left(0.2561\tau -0.2972\right)}^{2}}\\ -0.1262\;\cos\left(1.75\left(-0.957\tau -0.6639\right)\right)e^{-0.5{\left(-0.957\tau -0.6639\right)}^{2}}\\ +0.0208\;\cos\left(1.75\left(0.6513\tau -0.0050\right)\right)e^{-0.5{\left(0.6513\tau -0.0050\right)}^{2}}\\ -0.3607\;\cos\left(1.75\left(0.7574\tau -0.8275\right)\right)e^{-0.5{\left(0.7574\tau -0.8275\right)}^{2}}\\ +1.7204\;\cos\left(1.75\left(-0.058\tau -0.3235\right)\right)e^{-0.5{\left(-0.058\tau -0.3235\right)}^{2}}\\ -0.1039\;\cos\left(1.75\left(-0.271\tau -0.5232\right)\right)e^{-0.5{\left(-0.271\tau -0.5232\right)}^{2}}\\ +1.5608\;\cos\left(1.75\left(-0.3176\tau -1.242\right)\right)e^{-0.5{\left(-0.3176\tau -1.242\right)}^{2}}\\ +0.3663\;\cos\left(1.75\left(-0.8974\tau -0.693\right)\right)e^{-0.5{\left(-0.8974\tau -0.693\right)}^{2}}\\ -0.0041\;\cos\left(1.75\left(-2.0010\tau -1.863\right)\right)e^{-0.5{\left(-2.0010\tau -1.863\right)}^{2}}\\ -0.1883\;\cos\left(1.75\left(0.61200\tau +0.813\right)\right)e^{-0.5{\left(0.61200\tau +0.813\right)}^{2}}, \end{array}$$

(17) $$\begin{array}{c} \hat{Y}\left(\tau \right)=0.0097\;\cos\left(1.75\left(1.0108\tau +0.8687\right)\right)e^{-0.5{\left(1.0108\tau +0.8687\right)}^{2}}\\ +0.6808\;\cos\left(1.75\left(-0.475\tau +0.1533\right)\right)e^{-0.5{\left(-0.475\tau +0.1533\right)}^{2}}\\ +1.3976\;\cos\left(1.75\left(-0.107\tau +1.5804\right)\right)e^{-0.5{\left(-0.107\tau +1.5804\right)}^{2}}\\ -0.5523\;\cos\left(1.75\left(-0.066\tau -0.3244\right)\right)e^{-0.5{\left(-0.066\tau -0.3244\right)}^{2}}\\ +0.2293\;\cos\left(1.75\left(0.3343\tau +0.1346\right)\right)e^{-0.5{\left(0.3343\tau +0.1346\right)}^{2}}\\ +0.8040\;\cos\left(1.75\left(0.5024\tau +0.8675\right)\right)e^{-0.5{\left(0.5024\tau +0.8675\right)}^{2}}\\ +0.1466\;\cos\left(1.75\left(-0.761\tau +1.5040\right)\right)e^{-0.5{\left(-0.761\tau +1.5040\right)}^{2}}\\ +0.9269\;\cos\left(1.75\left(0.3945\tau -1.1415\right)\right)e^{-0.5{\left(0.3945\tau -1.1415\right)}^{2}}\\ +0.0374\;\cos\left(1.75\left(0.9908\tau -1.2051\right)\right)e^{-0.5{\left(0.9908\tau -1.2051\right)}^{2}}\\ +0.1970\;\cos\left(1.75\left(-0.764\tau +0.2823\right)\right)e^{-0.5{\left(-0.764\tau +0.2823\right)}^{2}},\\ -0.0384\;\cos\left(1.75\left(0.1343\tau +1.1398\right)\right)e^{-0.5{\left(0.1343\tau +1.1398\right)}^{2}}\\ +0.0150\;\cos\left(1.75\left(0.7727\tau +2.2949\right)\right)e^{-0.5{\left(0.7727\tau +2.2949\right)}^{2}}\\ -0.0024\;\cos\left(1.75\left(-0.829\tau +0.0417\right)\right)e^{-0.5{\left(-0.829\tau +0.0417\right)}^{2}}\\ +0.3144\;\cos\left(1.75\left(-0.365\tau +1.4552\right)\right)e^{-0.5{\left(-0.365\tau +1.4552\right)}^{2}}\\ -1.1990\;\cos\left(1.75\left(0.2513\tau -1.1402\right)\right)e^{-0.5{\left(0.2513\tau -1.1402\right)}^{2}}\\ +0.1784\;\cos\left(1.75\left(0.0640\tau -0.1835\right)\right)e^{-0.5{\left(0.0640\tau -0.1835\right)}^{2}}\\ +1.3200\;\cos\left(1.75\left(0.0134\tau -0.5702\right)\right)e^{-0.5{\left(0.0134\tau -0.5702\right)}^{2}}\\ -0.0002\;\cos\left(1.75\left(1.5840\tau -1.8226\right)\right)e^{-0.5{\left(1.5840\tau -1.8226\right)}^{2}}\\ -0.8039\;\cos\left(1.75\left(0.2124\tau +0.2349\right)\right)e^{-0.5{\left(0.2124\tau +0.2349\right)}^{2}}. \end{array}$$

(18) $$\begin{array}{c} \hat{Z}\left(\tau \right)=0.607\;\cos\left(1.75\left(0.1112\tau +1.3610\right)\right)e^{-0.5{\left(0.1112\tau +1.3610\right)}^{2}}\\ -0.0384\;\cos\left(1.75\left(0.1343\tau +1.1398\right)\right)e^{-0.5{\left(0.1343\tau +1.1398\right)}^{2}}\\ +0.0150\;\cos\left(1.75\left(0.7727\tau +2.2949\right)\right)e^{-0.5{\left(0.7727\tau +2.2949\right)}^{2}}\\ -0.0024\;\cos\left(1.75\left(-0.829\tau +0.0417\right)\right)e^{-0.5{\left(-0.829\tau +0.0417\right)}^{2}}\\ +0.3144\;\cos\left(1.75\left(-0.365\tau +1.4552\right)\right)e^{-0.5{\left(-0.365\tau +1.4552\right)}^{2}}\\ -1.1990\;\cos\left(1.75\left(0.2513\tau -1.1402\right)\right)e^{-0.5{\left(0.2513\tau -1.1402\right)}^{2}}\\ +0.1784\;\cos\left(1.75\left(0.0640\tau -0.1835\right)\right)e^{-0.5{\left(0.0640\tau -0.1835\right)}^{2}}\\ +1.3200\;\cos\left(1.75\left(0.0134\tau -0.5702\right)\right)e^{-0.5{\left(0.0134\tau -0.5702\right)}^{2}}\\ -0.0002\;\cos\left(1.75\left(1.5840\tau -1.8226\right)\right)e^{-0.5{\left(1.5840\tau -1.8226\right)}^{2}}\\ -0.8039\;\cos\left(1.75\left(0.2124\tau +0.2349\right)\right)e^{-0.5{\left(0.2124\tau +0.2349\right)}^{2}}. \end{array}$$

Systems (16)–(18) are implemented to solve the nonlinear SIR dengue fever system given in system (1) using the MWNN-GA-IPA and the acquired results are plotted in Figures 2–4.  Figure 2 shows the set of best weights and comparison of the best obtained results with the Runge–Kutta numerical results. It is seen that the proposed and reference results overlapped each other for $\hat{X}\left(\tau \right),$$\hat{Y}\left(\tau \right)$, and $\hat{Z}\left(\tau \right)$ classes to solve the nonlinear SIR dengue fever system. The plots of the AE for $\hat{X}\left(\tau \right),$$\hat{Y}\left(\tau \right)$, and $\hat{Z}\left(\tau \right)$ classes to solve the nonlinear SIR dengue fever system are reported in Figure 3. For the $\hat{X}\left(\tau \right)$ class, $\hat{Y}\left(\tau \right)$ class, and $\hat{Z}\left(\tau \right)$ class, the AE best values lie about 10^−6^–10^−8^, 10^−3^–10^−5^, and 10^−4^–10^−6^, and the AE mean values lie around 10^−1^-10^−2^, 10^−2^-10^−3^, and 10^−3^-10^−4^, respectively. The performance plots of the E-VAF and T.I.C indices for each class of the nonlinear SIR dengue fever system are plotted in Figure 4. For $\hat{X}\left(\tau \right)$ category, the best E-VAF, M.A.D, and T.I.C values lie around 10^−6^–10^−8^, 10^−5^-10^−6^, and 10^−9^-10^−10^. For $\hat{Y}\left(\tau \right)$ category, the best E-VAF, M.A.D, and T.I.C values lie around 10^−5^-10^−6^, 10^−3^-10^−4^, and 10^−8^-10^−9^. Similarly, for $\hat{Z}\left(\tau \right)$ class, the best E-VAF, M.A.D, and T.I.C values lie around 10^−3^-10^−4^, 10^−4^-10^−5^, and 10^−9^-10^−10^.

The graphical representations of the statistical trials along with the values of histograms are shown in Figures 5 and 6 for each class of nonlinear SIR dengue fever system. The convergence based on the E-VAF, M.A.D, and T.I.C operators is accomplished for independent trials to the nonlinear SIR dengue fever system. The achieved results from MWNN-GA-IPA are calculated satisfactory based on the T.I.C, M.A.D, and E-VAF operators.

For the accurateness and precision measures, statistical studies are provided in Tables 2–4 to solve each class of the nonlinear SIR dengue fever using the operatives minimum (Min), S.I range, maximum (Max), standard deviation (S.T.D), and median. The Min and Max standards show the best results and poorest results in the 100 executions. For *X*(*τ*) category, the Min, Max, median, S.I range, and S.T.D values lie around 10^−7^–10^−12^, 10^−1^-10^−2^, 10^−5^–10^−7^, 10^−5^-10^−6^, and 10^−1^-10^−2^, respectively. For the category *Y*(*τ*), the Min, Max, median, S.I range, and S.T.D values lie around 10^−4^-10^−5^, 10^−2^-10^−3^, 10^−4^-10^−5^, 10^−6^-10^−7^, and 10^−3^-10^−4^, respectively. Likewise, the Min, Max, median, S.I range, and S.T.D values for the category *Z*(*τ*) lie around 10^−5^–10^−11^, 10^−2^-10^−3^, 10^−4^–10^−7^, 10^−6^-10^−7^, and 10^−2^-10^−3^, respectively. These calculated presentations found the worth and value of the proposed MWNN-GA-IPA to solve the nonlinear SIR dengue fever system. One can establish through the achieved results that the MWNN-GA-IPA is stable and precise.

The global performance of the operators [G-M.A.D], [G-T.I.C], and [G-E.VAF] for 100 trials of MWNN-GA-IPA is plotted in Table 5 to solve each category of the nonlinear SIR dengue fever system. The global-based mean [G-M.A.D], [G-T.I.C], and [G-E.VAF] values are found to be 10^−4^-10^−5^, 10^−8^-10^−9^, and 10^−5^–10^−7^, whereas the global values of the S.I Range lie in the interval 10^−6^-10^−7^, 10^−10^-10^−11^, and 10^−6^-10^−7^ for each category of the nonlinear SIR dengue fever system. The close optimal outcomes acquired by the global measures approve the accurateness, correctness, and precision of MWNN-GA-IPA.

## 4. Conclusions

The current investigations are linked to design a neural network based on Morlet wavelet (MWNN) function for solving the nonlinear SIR dengue fever system based on dengue infection using the optimization procedures of global and local search approaches, i.e., GA-IPA. The nonlinear SIR dengue fever system is capable to evaluate through GA-IPA using the layer arrangement of Morlet wavelet neural networks taking 10 neurons. The overlapped results through MWNN-GA-IPA and the reference results show the good accuracy level to solve the nonlinear SIR dengue fever system based on dengue infection. The performance measures based on T.I.C, M.A.D, and E-VAF have been calculated satisfactorily. The statistical assessments for 100 independent trials using MWNN-GA-IPA in terms of minimum, S.I range, median, standard deviation, and maximum operatives further validate the worth and correctness of the proposed MWNN-GA-IPA. Furthermore, statistics analysis has been performed in the case of SIR dengue fever model based on dengue infection.

In future, the proposed MWNN-GA-IPA is proficient to solve the biological nonlinear systems, singular higher order nonlinear systems, and fluid dynamic systems.

## Figures and Tables

**Figure 1:** Structure of the present approach to solve the nonlinear SIR dengue fever system.

**Figure 2:** Best weight vector set and result comparison for each class of nonlinear SIR dengue fever system. (a) Best weights of *X*(*τ*) for 10 neurons. (b) Best weights of *Y*(*τ*) for 10 neurons. (c) Best weights of *Z*(*τ*) for 10 neurons. (d) Comparison for *X*(*τ*) class. (e) Comparison for *Y*(*τ*) class. (f) Comparison for *Z*(*T*) class.

**Figure 3:** AE values for each class of the nonlinear SIR dengue fever system. (a) AE for *X*(*τ*) class. (b) AE for *Y*(*τ*) class. (c) AE for *Z*(*τ*) class.

**Figure 4:** Performance of the E-VAF, M.A.D, and T.I.C operators for solving each class of the nonlinear SIR dengue fever system. (a) Performance for each class of the nonlinear SIR system.

**Figure 5:** Convergence of T.I.C plots along with the histogram using MWNN-GA-IPA to solve each class of the nonlinear SIR dengue fever system. (a) T.I.C for each class of the nonlinear SIR system. (b) Histogram for *X*(*τ*) class. (c) Histogram for *Y*(*τ*) class. (d) Histogram for *Z*(*τ*) class.

**Figure 6:** Convergence of M.A.D and E-VAF plots along with the histogram using MWNN-GA-IPA to solve each class of the nonlinear SIR dengue fever system. (a) Histogram for *X*(*τ*) class. (b) Histogram for *Y*(*τ*) class. (c) Histogram for *Z*(*τ*) class. (d) E-VAF for each class of the nonlinear SIR system. (e) Histogram for *X*(*τ*) class. (f) Histogram for *Y*(*τ*) class. (g) Histogram for *Z*(*τ*) class.

**Table 1:** Optimization performance taking the MWNN-GA-IPA for the nonlinear SIR dengue fever system.

**Start of GA**
**Inputs:** the chromosomes are characterized with the same system element as
*W* = [*v*, *w*, *u*]
**Population:** the chromosomes set is written as
*W*_*X*_=[*v*_*X*_, *ω*_*X*_, *u*_*X*_], *W*_*Y*_=[*v*_*Y*_, *ω*_*Y*_, *u*_*Y*_] and
**Output:** global values of the weight are represented as *W*_GA-Best_
**Initialization:** for the selection of chromosomes, select the weight vector values. **Fit evaluation:** modify the values of fitness “*e*” in population “*P*” for each vector with the use of systems 4–8
(i) **Stopping criteria:** terminate when [*e* = 10^−21^], [Generations = 55], [StallLimit = 140], [PopSize = 285], and [TolFun = TolCon = 10^−21^]
Move to **storage**
**Ranking:** rank individual weight vector in population using the values of the fitness
**Storage:** save *W*_GA-Best_, iterations, time, *e,* and count of function for the presence of GA
**End of GA**
**IPA starts**
**Inputs:** start point: *W*_GA-Best_
**Output:***W*_GA-IPA_ shows the best weight values of GA-IPA
**Initialize:***W*_GA-Best_, iterations, assignments, and other values
**Terminate:** stop, when [*e* = 10^−20^], [Iterations = 750], [MaxFunEvals = 267000], [TolCon = TolX = 10^−22^], and [TolFun = 10^−22^] achieved.
**Evaluation of fitness:** compute *W* and *e* using equations (8)–(12)
**Amendments:** adjust “fmincon” for IPA, compute *e* of better-quality of ‘W' using systems 4–8
**Accumulate:** transmute *W*_GA-IPA_, *e,* function counts, iterations, and time for the existing IPA runs
**IPA process ends**

**Table 2:** Statistical presentations of the nonlinear SIR dengue fever system for the category *X*(*τ*).

*τ*	*X*(*τ*)				
	Min	Max	Median	S.I range	S.T.D
0	4.0423220*E* − 12	9.9990000*E* − 01	2.2132198*E* − 07	3.3825540*E* − 06	2.9955460*E* − 01
0.1	1.8562196*E* − 08	9.9800585*E* − 01	2.2575664*E* − 06	9.2252690*E* − 06	3.1917267*E* − 01
0.2	1.1989577*E* − 08	9.9570595*E* − 02	2.8147596*E* − 06	7.3089931*E* − 06	3.1842462*E* − 02
0.3	3.2594992*E* − 07	9.9360942*E* − 01	3.6204945*E* − 06	5.6263588*E* − 06	3.1769837*E* − 01
0.4	9.7767938*E* − 08	9.9151010*E* − 01	5.4797252*E* − 06	5.1357097*E* − 06	3.1697503*E* − 01
0.5	3.2511304*E* − 06	9.8940563*E* − 02	8.1700536*E* − 06	7.3575618*E* − 06	3.1625439*E* − 02
0.6	2.8132523*E* − 06	9.8729376*E* − 01	1.1797241*E* − 05	1.1757718*E* − 05	3.1554735*E* − 01
0.7	6.9767773*E* − 07	9.8517226*E* − 01	1.5987828*E* − 05	9.1401060*E* − 06	3.1478449*E* − 01
0.8	6.3270889*E* − 06	9.8303897*E* − 02	2.0912004*E* − 05	1.0215585*E* − 05	3.1411641*E* − 02
0.9	4.5794286*E* − 06	9.8089357*E* − 01	2.5581289*E* − 05	9.6963771*E* − 06	3.1339004*E* − 01
1	3.0336439*E* − 06	9.7981727*E* − 01	3.1364852*E* − 05	1.1245408*E* − 05	3.1271044*E* − 02

**Table 3:** Statistical presentations of the nonlinear SIR dengue fever system for the category *Y*(*τ*).

*τ*	*Y*(*τ*)				
	Min	Max	Median	S.I range	S.T.D
0	4.7826156*E* − 05	1.2441636*E* − 03	5.3999940*E* − 04	2.1685104*E* − 07	1.9190429*E* − 04
0.1	2.2617648*E* − 04	3.1953335*E* − 03	5.3868377*E* − 04	2.2227911*E* − 06	6.0207993*E* − 04
0.2	2.4551957*E* − 04	5.1214677*E* − 03	5.3800062*E* − 04	2.9618951*E* − 06	1.3159469*E* − 03
0.3	2.1066905*E* − 04	7.0066945*E* − 03	5.3756084*E* − 04	2.1655938*E* − 06	2.0394513*E* − 03
0.4	1.7704587*E* − 04	8.9185145*E* − 03	5.3809794*E* − 04	1.9832062*E* − 06	2.7655709*E* − 03
0.5	1.7527548*E* − 04	1.0862314*E* − 02	5.3919348*E* − 04	1.6099165*E* − 06	3.4944298*E* − 03
0.6	1.5351687*E* − 04	1.2834137*E* − 02	5.4066226*E* − 04	1.7106495*E* − 06	4.2264704*E* − 03
0.7	4.2598412*E* − 05	1.4831228*E* − 02	5.4286714*E* − 04	2.3156731*E* − 06	4.9614134*E* − 03
0.8	1.2432002*E* − 04	1.6851840*E* − 02	5.4585539*E* − 04	3.3573941*E* − 06	5.6986905*E* − 03
0.9	1.2880654*E* − 04	1.8894845*E* − 02	5.4928063*E* − 04	3.3031846*E* − 06	6.4404297*E* − 03
1	9.7394166*E* − 05	2.0992829*E* − 02	5.5344362*E* − 04	2.9146189*E* − 06	7.1876800*E* − 03

**Table 4:** Statistical presentations of the nonlinear SIR dengue fever system for the category *Z*(*τ*).

*τ*	*Z*(*τ*)				
	Min	Max	Median	S.I range	S.T.D
0	2.7359906*E* − 11	6.0293074*E* − 02	2.1020438*E* − 07	1.4892650*E* − 06	1.6947015*E* − 02
0.1	1.2779827*E* − 06	6.0606789*E* − 02	1.7227698*E* − 05	2.9467734*E* − 06	1.8379946*E* − 02
0.2	9.8289161*E* − 07	6.0932383*E* − 02	3.4063897*E* − 05	4.1260050*E* − 06	1.8423547*E* − 02
0.3	7.8962744*E* − 06	6.1220946*E* − 02	5.0622682*E* − 05	2.7004041*E* − 06	1.8477633*E* − 02
0.4	2.8442743*E* − 05	6.1487380*E* − 02	6.6956094*E* − 05	1.7144321*E* − 06	1.8548676*E* − 02
0.5	4.3296911*E* − 05	6.1745495*E* − 02	8.3558913*E* − 05	2.8627209*E* − 06	1.8637956*E* − 02
0.6	6.4428148*E* − 05	6.2007841*E* − 02	1.0025700*E* − 04	3.3723574*E* − 06	1.8746689*E* − 02
0.7	7.8570024*E* − 05	6.2285742*E* − 02	1.1721379*E* − 04	3.3496552*E* − 06	1.8875847*E* − 02
0.8	8.0198804*E* − 05	6.2589332*E* − 02	1.3406477*E* − 04	3.9024126*E* − 06	1.9025869*E* − 02
0.9	4.5991286*E* − 05	6.2927739*E* − 02	1.5084468*E* − 04	2.3165808*E* − 06	1.9198331*E* − 02
1	4.4797926*E* − 05	6.3311235*E* − 02	1.6779808*E* − 04	4.5753017*E* − 06	1.9389410*E* − 02

**Table 5:** Global presentations for each category of the nonlinear SIR dengue fever system.

Category	[G-M.A.D]		[G-T.I.C]		[G-E.VAF]	
	Mean	S.I range	Mean	S.I range	Mean	S.I range
*X*(*τ*)	1.14673*E* − 05	7.46457*E* − 06	1.09132*E* − 09	5.61892*E* − 11	2.30930*E* − 06	1.16918*E* − 06
*Y*(*τ*)	5.42141*E* − 04	1.85278*E* − 07	3.86220*E* − 08	1.58454*E* − 10	6.26006*E* − 07	4.76894*E* − 07
*Z*(*τ*)	8.40963*E* − 05	2.85409*E* − 06	7.05895*E* − 09	2.03526*E* − 10	6.46250*E* − 05	1.58215*E* − 06

## Data Availability

This work is not based on any data.
